The article "Corner Detection of the Computer VR Microscope Image Based on the 3D Reconstruction Algorithm" was retracted in 2023. Reasons: signs of a paper mill; suspected computer-generated content; unreliable results or conclusions; concerns about the data.

# Corner Detection of the Computer VR Microscope Image Based on the 3D Reconstruction Algorithm

**DOI:** 10.1155/2022/8621103

**Published:** 2022-07-20

**Authors:** Junjun Huang

**Affiliations:** Fujian Vocational College of Agriculture, Fuzhou, Fujian 350119, China

## Abstract

In order to solve the problem of multisolution and ill-formedness of the 3D reconstruction method of a single image (purpose), the author proposes a microscope image segmentation algorithm based on the Harris multiscale corner detection. Separating complex engineering images into several simple basic geometric shapes, rebuild them separately to avoid the ill-conditioned solution problem of directly recovering depth information. In order to improve the registration accuracy of the corner-based image registration algorithm, the idea of multiresolution analysis was introduced into the classic Harris corner detection, and a gray intensity variation formula based on the wavelet transform was constructed, and a scale transformation characteristic was obtained so that the improved Harris corner detection algorithm is invariant to rotation, translation, and scale. Experimental results show that after reconstruction, the error between the length of the object measured based on the point cloud data and the actual length of the object is small, and both remain within the error range of 3 mm. The experiment verifies the fast, accurate, and stable characteristics of the improved algorithm.

## 1. Introduction

80% of the information that humans understand and explore the world is the visual information obtained by the eyes. With the rapid development of modern computer technology, people have begun to try to make computers have visual functions similar to those of humans, replacing human eyes with cameras, capturing images through cameras, and then using computers to analyze and understand the captured images; the output of advanced visual information helps us to recognize and understand the world faster and better, resulting in the new discipline of computer vision [1].

3D reconstruction technology is one of the important branches of computer vision technology (Figure 1), and it is a popular research field combining computer vision and industrial measurement. Among them, in the fields of rapid design of industrial products, automatic detection and measurement, quality inspection and control, 3D printing, and other fields, the demand for fast, accurate, and convenient acquisition of 3D information on the surface of objects is increasing [2].

At present, structured light technology is the most reliable and effective technology to achieve the three-dimensional reconstruction of the object surface [3]. This technology first projects the structured light coding pattern onto the surface of the target object to be measured through a projector and then uses a camera to shoot the surface of the target object; the camera will capture the structured light image whose coding pattern is deformed due to the shape of the surface of the target object, decode the deformed structured light image, and then calculate the 3D point cloud data of the object surface based on the principle of triangulation so as to realize the three-dimensional reconstruction of the surface of the measured object. With the rapid development of science and technology, various fields hope to achieve the high-precision 3D reconstruction of the surface of high-speed moving objects; in order to achieve the 3D reconstruction of moving objects, only a single image can be used for 3D reconstruction; therefore, 3D reconstruction based on a single image has become an important research direction in the field of structured light technology.

## 2. Literature Review

Research on the application of the active structured light method in the detection of the three-dimensional topography of objects started in the 1970s. Huang et al. proposed a method for projecting slit structured light to identify polyhedra. With the development of structured light technology, projection modes have also been developed; in particular, the emergence of encoded structured light solves the limitation of additional geometric constraints. Coding structured light can be divided into temporal coding and spatial coding according to different coding methods. The time coding method uses the preprojected image to the surface of the object and then creates the code, so the complete final code pattern cannot be formed until all the patterns are completely projected, and the encoding is closely related to the projection position [4]. Li et al. projected a grayscale-encoded pattern with marked sinusoidal intensities onto the object surface, solving the problem of ambiguity of the projected signal at each different time [5]. Based on the use of *N*-ary, Tang et al. proposed a color-based projection scheme and established a reflection model, which contains *n*^*m*^ fringes in the RGB color space, and the number of fringe projections directly affects the measurement efficiency of the system [6]. In order to reduce the number of streaks, Pan and Zhu developed a hybrid system that can simultaneously fuse temporal and spatial encoding; the system has a fast processing speed and high measurement accuracy and can be applied to dynamic measurement; the projected structured light can be encoded according to the time axis; at the same time, it can also be encoded according to the spatial neighborhood points [7]. Gao et al. proposed a pseudorandom sequence; due to the uniqueness of the window, each different subsequence can find the absolute position in the whole sequence; it is widely used in spatial coding schemes. Spatial encoding can be regarded as a sequence set based on pseudorandom numbers; the encoding pattern is generated by a Hamming window or an *N*-dimensional Euler path; the feature positions are determined by observing the line colors stored in the same window [8]. In 1998, Peng et al. proposed an orthogonal vertical grid color coding, which uses the peak concentration to detect the intersection, and at the same time, it converts the color from the RGB space to the HSI space for encoding, but in the decoding process, due to the different reflection of illuminance, the H channel is sensitive, which leads to new problems [9]. Feng et al. proposed an encoding scheme combining traditional stripes and multislit structured light, which again improved the measurement accuracy [10].

For the 3D reconstruction of a single 2D engineering geometry, the author proposes a new research method, which avoids the ill-conditioned solution problem of traditional methods. Firstly, using the microscope image segmentation algorithm based on the Harris multiscale corner detection, a complex combined graph is separated into several simple primitives, and then each primitive is reconstructed in 3D, which not only reduces the complexity of the reconstruction algorithm but also improves the real-time performance. The improved corner detection algorithm can obtain corners at different scales, thus overcoming the possible corner information loss, the position offset and susceptibility to noise in the Harris corner detection of a single scale, and the extraction of false corners and other problems. Secondly, the relationship between image matching and image corner matching is studied; the algorithm takes the corner as the feature point of the image and uses four indicators, such as the corner value, the number of neighborhood corners, the distance between the corners, and the consistency of parameters; filter the set of corner points step by step; the unmatched corners are effectively eliminated; the matching accuracy is ensured, and at the same time, the heavy calculation of template matching in the traditional algorithm is avoided, and the matching speed is greatly improved.

## 3. Research Methods

### 3.1. Harris Multiscale Corner Detection Principle and Corner Extraction

#### 3.1.1. The Principle and Limitation of the Classic Harris Corner Detection

The corner point is an important image feature point, which contains rich two-dimensional structural information; in the fields of feature-based image registration, shape recognition, and three-dimensional reconstruction, corner point extraction is of great significance. The most representative corner detection algorithm is the Harris corner detection algorithm [11]. The Harris operator is a signal-based corner feature extraction operator proposed by Harris and Stephens; it has the characteristics of simple calculation, uniform and reasonable extraction of corner features, quantitative extraction of feature points, and a stable operator. The processing process of the classic Harris corner detection algorithm is expressed as the following formulas:

(1) $$\begin{array}{c} M=G\left(\tilde{s}\right)⊗\left[\begin{array}{cc} g_{x}^{2} & g_{x}g_{y}\\ g_{x}g_{y} & g_{x}^{2} \end{array}\right],\\ R=\det\left(M\right)-k\cdot {\text{tr}}^{2}\left(M\right),\;k=0.04, \end{array}$$

where *g*_*x*_ and *g*_*y*_ are the gradients in the *x* and *y* directions, respectively, $G\left(\tilde{s}\right)$ is the Gaussian template, det is the determinant of the matrix, tr is the straight trace of the matrix, *k* is a constant, and *R* represents the interest value of the corresponding pixel in the graph. If the interest value of a certain pixel is in the largest neighborhood and is greater than the threshold (*R*_0_), the pixel is called a corner, and the corresponding interest value is called a corner value. Although the Harris corner detection is a classic algorithm, it has the following shortcomings. (1) Since corners can only be detected at a single scale, nonmaximum suppression is performed on the corner metric to determine local maxima, and the extraction effect depends on the setting of the threshold. The threshold will lose corner information, and if the threshold is small, false corners will be extracted. Therefore, the lack of scale function makes the positioning accuracy of the algorithm poor, and it may also miss some actual corner points, which are also sensitive to noise. (2) The Harris corner detection uses a Gaussian smoothing function with an adjustable window, but the size of the Gaussian window is not easy to control. If the window is small, many false corners will appear due to the influence of noise. If the window is larger, the position of the corner points will be greatly offset due to the rounded corner effect of the convolution, and the calculation amount will be increased [12]. (3) Smoothing the image with an infinitely smooth Gaussian function will result in the loss of corner information due to oversmoothing.

#### 3.1.2. Improved Harris Multiscale Corner Detection

In view of the problems existing in the Harris corner detection algorithm, the idea of multiresolution analysis is introduced into the algorithm so that the Harris algorithm has the characteristics of multiscale detection of corners. This is based on the following principles. In the Harris algorithm, *g*_*x*_ and *g*_*y*_ reflect the gray level change direction of each pixel of the image, and if the brightness of pixel (*x*, *y*) changes sufficiently in all directions, it is extracted as a corner [13]. The wavelet Ψ_*u*,*s*_ (*t*) is a function with a mean of 0, and the wavelet transform of the signal *g* is

(2) $$\begin{array}{c} W_{g}\left(u,s\right)=g*\Psi_{u,s}\left(t\right)=\int_{-\infty }^{+\infty }\;g\left(t\right)\Psi_{u,s}\left(t\right)dt. \end{array}$$

It measures the variation of the signal within a neighborhood centered on *u* and whose length is proportional to *s*. And if the wavelet has a first-order or *n*-order vanishing moment, the wavelet transform is a multiscale differential operator [14]. Therefore, use the wavelet transform of the image to redefine the gray intensity change formula of the image, that is, the following formula:

(3) $$\begin{array}{c} E_{u,y}\left(x,y\right)=S_{2^{j}}{\left(uW_{2^{j+1}}^{1}f+vW_{2^{j+1}}^{2}+f\right)}^{2}=\left(S_{2^{j}}u^{2}{\left(W_{2^{j+1}}^{1}+f\right)}^{2}+2uvW_{2^{j+1}}^{1}fW_{2^{j+1}}^{2}f+v^{2}{\left(W_{2^{j+1}}^{2}+f\right)}^{2}\right)=Au^{2}+2Cuv+Bv^{2}=\left(u,v\right)\left(\begin{array}{cc} A & C\\ C & B \end{array}\right){\left(u,v\right)}^{T}. \end{array}$$

Among them, *W*_2^*j*+1^_^1^*f* and *W*_2^*j*+1^_^2^*f*, respectively, represent the wavelet transform of the image *f* in the *x* and *y* directions, that is, the following formulas:

(4) $$\begin{array}{c} W_{2^{j+1}}^{1}f=S_{2^{j}}^{d}f⊗\left(G_{j},D\right),\\ W_{2j+1}^{2}f=S_{2^{j}}^{d}f⊗\left(D,G_{j}\right). \end{array}$$

And *S*_2^*j*^_ represents the smoothing operator, so we have

(5) $$\begin{array}{c} A=S_{2^{j}}\left[\left(W_{2^{j+1}}^{1}\right)\right]={\left(W_{2^{j+1}}^{1}\right)}^{2}⊗\left(H_{j},H_{j}\right),\\ B=S_{2^{j}}\left[{\left(W_{2^{j+1}}^{2}\right)}^{2}\right]=\left(W_{2^{j+1}}^{2}\right)⊗\left(H_{j},H_{j}\right),\\ C=S_{2^{j}}\left[\left(W_{2^{j+1}}^{1}W_{2^{j+1}}^{2}\right)\right]=\left(W_{2^{j+1}}^{1}W_{2^{j+1}}^{2}\right)⊗\left(H_{j},H_{j}\right). \end{array}$$

⨂ is the convolution operation, *H* and *G* are the low-pass and high-pass filters, respectively, *D* is the Dirac filter, and *H*_*j*_ and *G*_*j*_ represent the insertion of 2^*j*^ − 1 zeros between the filter coefficients of *H* and *G*, respectively. In this way, the autocorrelation matrix of pixel point (*x*, *y*) at scale *j* + 1 is obtained as follows:

(6) $$\begin{array}{c} M_{2}^{j+1}=\left(\begin{array}{cc} A & C\\ C & B \end{array}\right). \end{array}$$

It is worth noting that Equation (3) not only reflects the gray intensity change of each pixel but also reflects the information of the scale space change, which enables corner detection at different scales [15]. At the same time, the central B-spline function with low-pass characteristics is selected as the smoothing function; it can make up for the insufficiency of the Gaussian function window that is difficult to control and oversmooth in the Harris algorithm and enhance the corner detection performance.

Like the Harris algorithm, if the two eigenvalues *λ*_1_ and *λ*_2_ of the autocorrelation matrix are large enough, the pixel is detected as a corner point. In order to avoid the eigenvalue decomposition of the matrix *M*_2_^*j*−1^, the corner response function (CRF) under the scale *s* = 2^*j*+1^ is defined as the following formula:

(7) $$\begin{array}{c} C_{2}^{j+1}\left(x,y\right)=\det\left(M_{2}^{j+1}\right)-k{\left(\text{trace}\left(M_{2}^{j+1}\right)\right)}^{2}. \end{array}$$

Among them, det(*M*_2_^*j*+1^) = *λ*_1_*λ*_2_ = *AB* − *C*^2^, trace (*M*_2_^*j*+1^) = *λ*_1_ + *λ*_2_ = *A* + *B*, and *k* is a given constant ranging from 0.04 to 0.06. At this time, the noise is eliminated by setting a threshold value, and nonmaximum value suppression is performed to determine the corner points; that is, the pixel point (*x*, *y*) that satisfies *C*_2_^*j*+1^(*x*, *y*) > *T* is determined as the corner point. The new Harris multiscale corner detection method obtains corner information at multiple scales, reducing the restriction of threshold setting on corner extraction. Usually, the detection operator of small-scale parameters can detect subtle changes in the gray level and reflect more singular point information, but it is more sensitive to noise. The detection operator of large-scale parameters can detect rough changes in the gray level and reflect sharply changing singular points, and it has strong suppression of noise. Therefore, the multiscale Harris corner detection achieves precise localization at small scales and removal of falsehoods and preservation of truth at large scales [16]. After the Harris multiscale corner detection, the author proposes the following “fine-to-coarse” method to accurately screen corners at different scales.

Firstly, for the modulus maximum point *P*_*j*_ that appears in the 2^*j*^ and *j* = 1 scales, the corner response function *C*_2_^*j*^(*x*_*j*_, *y*_*j*_) is calculated; when its value exceeds the threshold *T*_*j*_, this point is extracted as a candidate corner point. Selecting the scales of 2^*j*^ and *j* = 1 is to use the wavelet transform to accurately locate the corners at small scales to determine the position of the corners; therefore, all corners can be included in this step.

Secondly, at the scale of 2^*j*+1^, observe whether there is a maximum point in *C*_2_^*j*+1^(*x*_*j*_, *y*_*j*_) near the candidate corner point *P*_*j*_ obtained in the previous step; if it exists, it is determined that the point is a corner point; if not, the point can be eliminated from the candidate corner points.

#### 3.1.3. Analysis of the Experimental Results of the Algorithm

In the experiment, the central B-spline function with low-pass characteristics is selected as the smooth function of the corner detection operator because the function has good approximation ability and compact support and other excellent properties. When the order of the B-spline function tends to infinity, it converges to the Gaussian function, and its derivative converges to the derivative of the Gaussian function. The statistics in Table 1 fully demonstrate the superiority of the improved algorithm in terms of localization, effectiveness, and noise immunity in extracting corners [17].

### 3.2. Body Segmentation Algorithm Based on Corner Detection

The basic idea of the adopted body segmentation algorithm is as follows. The basic geometric primitives in the field of engineering drawing are as follows: cylinder, cuboid, sphere, wedge, cone, etc. If all kinds of basic primitives contained in complex two-dimensional engineering drawings can be detected, it is easy to segment them. The process of detecting the basic primitives from the combined image is actually an image registration process; that is, the images to be separated are sequentially registered with the standard images of the basic shapes. Based on this, the categories and positions of the basic primitives contained in the image to be separated are determined. But there are two deficiencies in the common matching algorithms based on image features. First, the matching accuracy of the algorithm is not high and the stability is not good. Since the matching algorithm only uses a small part of the information of the image, the matching result is easily affected by factors such as noise and image information distribution, and it is highly dependent on the accuracy and stability of the feature points. Second, the matching search speed of feature points still needs to be improved [18]. Most of the matching algorithms use the template correlation method to perform the ergodic matching search; therefore, the algorithm is computationally expensive and slow.

Aiming at the above two shortcomings, the author proposes a new matching algorithm based on corner detection. Firstly, the feature points of the image are extracted by the multiscale Harris operator with less computational complexity and better stability, and the corner sets of the reference image and the image to be matched are obtained, respectively. Then, according to the relationship between the matching of corner sets, the image corners are gradually screened from three aspects: alignment, the number of neighborhood corners, and the distance between corners; due to the instability of the corner detection algorithm and other factors, the image matching is affected, and finally, an accurate and stable matching corner set is obtained [19].

Figure 2 is a graph in which the cylinder is rotated 45 degrees clockwise, and it can also be regarded as a projection graph obtained from different viewing angles for the same three-dimensional entity, which requires the registration algorithm to map them as an entity, and the improved Harris multiscale corner detection algorithm has rotation invariance, translation invariance, and scale invariance, which solves the problem of “many” versus “one” very well [18].

When matching the feature points of two images, choosing an appropriate similarity algorithm can improve the matching efficiency and accuracy. The alignment degree of the corner point pair (CPAM) is defined to determine the matching point pair; that is, on the basis of the corner point and its gradient information extracted by the Harris multiscale corner point detection algorithm, the approximate rotation angle is obtained according to the angle histogram statistics, the feature submaps centered on the corners are extracted from the two images to be registered, and the alignment of all these feature submaps is calculated.

#### 3.2.1. Angle Histogram for Corner Point Pairs

Assuming that there are two images *f*_1_(*x*, *y*) and *f*_2_(*x*, *y*) to be registered, the extracted corner sets are *P*_*f*1_ = {*p*_*i*_ = (*p*_*x*_^*i*^, *p*_*y*_^*i*^)}_*i*=1,2,⋯,*N*_ and *P*_*f*2_ = {*q*_*j*_ = (*q*_*x*_^*i*^, *q*_*y*_^*i*^)}_*j*=1,2,⋯,*N*_, respectively, where *θ*_*p*1_ and *θ*_*q*1_ are the gradient vector directions of *p*_*i*_ and *q*_*j*_, respectively. Define the angle histogram *H* (*θ*) of the corner point pair, indicating the number of the corresponding corner point pairs in *P*_*f*1_ and *P*_*f*2_ when the angle difference is *θ*. The *θ* value when *H* (*θ*) takes the maximum value also represents the rotation angle between the images *f*_1_(*x*, *y*) and *f*_2_(*x*, *y*). In order to improve the accuracy of the algorithm, modify *H* (*θ*).

The rotation angle *θ* between images can be estimated by searching for the angle corresponding to the maximum value of (*θ*). This method of using statistics to obtain the rotation angle has the advantages of the small amount of calculation and accurate calculation.

#### 3.2.2. Alignment of Corner Point Pairs

The alignment of the corner point pair is defined as the following formula:

(8) $$\begin{array}{c} \bar{\text{CPAM}}\left(p,q_{j},\theta \right)=\frac{1}{100\cdot \text{CI}\left(I_{1},I_{2}\right)+1}. \end{array}$$

In the formula, *I*_1_ and *I*_2_ are the corresponding two feature submaps, and CI is the interaction variance of the two feature submaps, which reflects the stability of the corresponding gray levels of the two feature submaps. For the corner point *q*_*j*_ in the image *f*_2_(*x*, *y*) to be registered, its matching corner point *p* is determined in the corner point set *pf*_1_ of another image *f*_1_(*x*, *y*) to be registered. If and only if *p* and *q*_*j*_ satisfy the following conditions, {*p*⇔*q*_*j*_} becomes a candidate matching point pair.

(9) $$\begin{array}{c} \left|\theta_{i,j}-\theta \right|<5^{\circ },\;\theta_{i,j}=\theta_{p}-\theta_{qj},\\ \bar{\text{CPAM}}\left(p,q_{j}\right)=\underset{p_{i}\in {pf}_{1}}{\max}\;\bar{\text{CPAM}}\left(p_{i},q_{j}\right),\\ \bar{\text{CPAM}}\left(p,q_{j}\right)>T_{a},\;T_{a}\text{ is the threshold}. \end{array}$$

In the formula, *θ*_*p*_ represents the gradient direction of the corner point *P*, and the threshold (*T*_*a*_) is the mean of the variance of the two feature submaps. Finally, the candidate matching point pairs are linearly weighted to eliminate the wrong matching point pairs, and a subset of matching corner point pairs is initially obtained. It should be noted that the corner points in subsets *C*_1_ and *C*′_1_ whose corner point values are matched do not necessarily correspond one-to-one; that is, the number of corner points contained in *C*_1_ and *C*′_1_ may be different.

#### 3.2.3. Neighborhood Corner Matching

If images A and B match, the two matching corners on them should have the same number of corners in the same neighborhood. Therefore, the corner points in *C*_1_ and *C*′_1_ that do not meet this condition are eliminated through the number of neighborhood corner points matching, and new corner point sets *C*_1_ = {*c*_1_, *c*_2_, ⋯, *c*_*g*_} and *C*_2_′ = {*c*_1_′, *c*_2_′, ⋯, *c*_*h*_′} are obtained. Similarly, the number of corner points in *C*_2_ and *C*′_2_ may also be different [20].

#### 3.2.4. Corner Spacing Match

If images A and B match, the distances between the corresponding two corner points and the other corresponding corner points in their respective neighborhoods should be the same; therefore, the corner point spacing matching is to further eliminate the corner points in *C*_2_ and *C*′_2_ that do not meet this condition and get new subsets *C*_3_ and *C*′_3_. The specific operations are as follows. Let *c*_*i*_ and *c*′_*i*_ be a pair of corner points that have satisfied the matching of the value of corner points and the matching of the number of neighborhood corner points. Let the number of neighborhood corner points be *p*, and the distances from *c*_*i*_ and *c*′_*i*_ to the corner points of their neighborhoods are arranged in descending order as {*d*_1_, *d*_2_, ⋯, *d*_*p*_} and {*d*′_1_, *d*′_2_, ⋯, *d*′_*p*_}; if {*d*_1_, *d*_2_, ⋯, *d*_*p*_} and {*d*′_1_, *d*′_2_, ⋯, *d*′_*p*_} are equal in one-to-one correspondence within the allowable deviation range, *c*_*i*_ and *c*′_*i*_ are considered to be matching corners; otherwise, they are not. After the above steps, the number of corner points contained in the two corner point sets (*C*_3_ and *C*′_3_) may still be inconsistent. For the convenience of calculation, the “one-to-one correspondence” or “one-to-many correspondence” corners can be directly eliminated so that *C*_3_ and *C*′_3_ contain the same number of corners, that is, *C*_3_ = {*c*_1_, *c*_2_, ⋯, *c*_*f*_} and *C*′_3_ = {*c*_1_′, *c*_2_′, ⋯, *c*′_*f*_}.

#### 3.2.5. Body Segmentation Algorithm Flow

After the above three steps of detection, it is possible to basically determine which basic geometric primitives are included in the two-dimensional graphics to be reconstructed and then determine the positional relationship between the basic geometric shapes included; these relationships are the basis for the BOOL operation on the reconstructed basic shape. The flow of the whole body segmentation algorithm is shown in Figure 3. When the final matching subset does not exist, it is necessary to expand the matching condition to continue the matching search, but the matching condition has a threshold; when the maximum search condition is reached and still no valid subset is obtained, it is considered that the image to be reconstructed does not have any valid subset and contains any of the basic shape classes.

## 4. Analysis of Results

For the combined graph shown in Figure 4(a), it is extremely difficult to reconstruct it directly in 3D, but if it is separated into several basic geometric shapes and then 3D reconstruction is carried out separately, a complex problem is solved.  Figure 4 is an example of a 3D reconstruction. Among them, Figure 4(b) shows the corner points extracted by the Harris multiscale corner point detection algorithm [21]; the extracted corner point sets are sequentially registered with the standard corner point subsets of various basic shapes in order to confirm the basic shape type contained in the 2D image to be reconstructed. Part of the shape may be occluded; as shown in Figure 4(b), a corner of the lower cuboid is covered by the middle cylinder, and sometimes, there will be more interference corners, such as the intersection of the middle cylinder and the two edges of the cuboid; the generated corners, for these cases, require the shape separation algorithm to appropriately relax the conditions when making matching criteria.  Figure 4(c) is the result of the shape separation algorithm, which is composed of two cylinders and a cuboid.

Taking the reconstruction of a cuboid as an example to illustrate the 3D reconstruction process of a single basic geometric body, because it is known that the type of the shape is a cuboid, in order to reconstruct its contour information in the three-dimensional space, it is necessary to know the dimensions of the length, width, and height of the cuboid and the coordinates of its centroid [22]. The centroid coordinates are easy to determine. Then, using the calculation result of the corner point histogram in Section 3.2, we can know the rotation angle of the cuboid in the reconstructed image relative to the standard shape, use the rotation angle to correct the cuboid in the image to be reconstructed, and then easily calculate the length, width, and height information according to the distance between the corresponding corner pairs. The rest of the geometry reconstruction process is similar.

The number of reconstructed point clouds proposed by the author is more than 15,000; in addition, as shown in Figure 5, the average error and standard deviation of the three-dimensional point cloud data statistics and the measurement results are compared; the average error and standard error can show that the author's reconstruction algorithm has high accuracy; after reconstruction, the length of the object measured based on the point cloud data and the actual length of the object have a small error, which are kept within the error range of 3 mm; through these experimental data, it is fully verified that the algorithm proposed by the author can effectively improve the accuracy of 3D reconstruction [23].

Finally, each reconstructed single shape is drawn in the three-dimensional space through the BOOL operation. The system is based on the VC++ 6.0 development platform through the embedded Open Inventor 3D graphics library for 3D data processing [24].

## 5. Conclusion

3D reconstruction based on a single image is one of the major challenges faced by human beings in basic and applied research, and there are still many difficulties that have not been satisfactorily resolved. The improved algorithm provides a new idea for the 3D reconstruction of engineering drawings, which is to separate the complex composite body into simple basic geometric shapes, then reconstruct them, respectively, and divide the reconstructed basic shapes according to their relative positions; the relationship performs BOOL operations to obtain the geometric entity model in the 3D space. The image registration algorithm based on the Harris multiscale corner detection is used in the separation algorithm; this algorithm is aimed at the classic Harris corner detection algorithm; the principle of multiscale detection can only be introduced for the drawbacks of single-scale detection so that the corner detection algorithm has rotation invariance, translation invariance, and scale invariance. The algorithm can also be widely used in other corner detection fields.

## Figures and Tables

**Figure 1:** 3D reconstruction algorithm.

**Figure 2:** The various rotation effects of the cylinder.

**Figure 3:** Flowchart of the body segmentation algorithm.

**Figure 4:** 3D reconstruction example.

**Figure 5:** Average error and standard deviation of 3D point cloud data statistics and measurement results.

**Table 1:** Statistics of the number of corner points.

Detector	Exact corner	Missing corner	Pseudocorner
Classic Harris algorithm	40	7	11
Improved algorithm	45	2	3

## Data Availability

The data used to support the findings of this study are available from the corresponding author upon request.
